# Walking and Activeness: The First Step toward the Prevention of Strokes and Mental Illness

**DOI:** 10.1155/2022/3440437

**Published:** 2022-03-14

**Authors:** Ning An, Jing Chuo

**Affiliations:** College of Physical Education, Taiyuan University of Technology, Taiyuan 030024, China

## Abstract

Physical activity, especially routine walking, is an imperative factor for the prevention of strokes, mental illness, and cardiovascular diseases (CVDs). The NIH (National Institute of Health) has also acknowledged walking as the most important factor of the stroke rehabilitation program. Many research studies are presented by physicians and researchers in the literature that highlight the positive impacts of walking on human health (physical and mental). This paper has the objective of studying the impact of regular walking, especially on mental illness, CVDs, and strokes. The C-reactive protein (CRP), P-selectin protein, and homocysteine biomarkers are considered to decide the improvement in the health of an individual with respect to CVDs and strokes. The other parameters considered for the recommendations of physicians and healthcare experts for mental health are PSS (perceived stress score) and ESS (Epworth sleepiness score) that control mental illness. The values are measured for the participating subjects before participating in the walking activity and after the end of the walking schedule to see the impact on individuals. The overall mental and physical health of an individual contributes to the chances of occurrence of CVDs, mental illness, and strokes in individuals aged between 40 years and 55 years, as per the study presented in this paper. The results show that the PSS and ESS scores are improved after the walking activity. Eventually, it improved recovery from many kinds of mental illness and also reduced the chances of strokes. Similarly, the levels of the biomarkers that determine the chances of an individual having CVD or stroke also improved. Walking can impact our overall health in many ways, however, in this paper, the focus is given to ailments, such as strokes, CVDs, and mental illness. The results show that stress and improper sleepiness can impact mental health negatively. The research outcome is measured by adding walking in a routine life so that every individual can get rid of many physical and mental ailments. The results presented in the paper reveal that the 90-day walking program has created a good impact on the health of individuals by improving their physical and mental health.

## 1. Introduction

A stroke is a medical emergency that occurs when a blood artery that supplies oxygen and nutrients to the brain is blocked, generally because of a blood clot [1]. Stroke symptoms include difficulty in walking, talking, and understanding, along with paralysis or numbness of the face, arm, or leg. Clinical manifestations include the stiffness or paralysis of the face, hand, or limb, along with trouble while walking, talking, and comprehending. In the United Kingdom, it is the third-largest risk factor for death rate and the main factor of acquired impairment. Every year, over 130,000 people experience their first stroke [2]. In addition to easily available pharmacological therapy for stroke prevention, stroke avoidance and rehabilitative treatments are necessary. Moreover, establishing such techniques is a major undertaking of 21^st^-century medicine. The role of physical exercise in lifestyle modification is of significant interest because of the sheer high morbidity, mortality, and huge burden of stroke-related comorbidities on patients and health care resources. The use of physical exercise is similar to a therapeutic method.

There is a lot of data to promote the use of endurance training in patients with risk factors, both quantitative and qualitative. In the rehabilitation of stroke victims, there is a huge amount of research that endorses the objective of maximum treatment outcomes. Indoor activities, such as playing computer games, watching Television, accessing computers, and staying in one spot for long periods of time, contribute to a sedentary lifestyle. It has a number of negative consequences for our bodies. Muscular endurance deteriorates, and nutrient composition decreases, causing bones to deteriorate [3]. Carbohydrates and lipids are tough for the body to break down. The circulatory system is harmed, the cells are inflamed, and there is a hormonal imbalance. Overweight, cardiovascular disease, high cholesterol, heart problems, stroke, metabolic disorders, hypoglycemia, malignancy, anxiety, stress, cancers, and other disorders connected with these maladies are all induced by physical inactivity [4]. To lower the chance of developing such diseases, one should adopt a healthier lifestyle and incorporate physical activity into one's daily routine [5].

The correlation between walking and cerebrovascular disease is complicated, and it interests doctors, physiotherapists, and epidemiologists to figure out all the factors that impact positively and negatively on such kinds of diseases. Physical inactivity was identified as one of the five key risk factors in stroke-related research, accounting for approximately more than 80% of the worldwide stroke incidence rates, as per the statistical data [6, 7]. Walking and physical activities are sharply promoted as a facet of stroke treatment programs and mental health improvement programs because of the rising pile of empirical studies demonstrating its advantages in the treatment of these diseases [8, 9]. This paper presents a comprehensive review of the studies on the relationship between physical exercise and CVD-related illnesses, including strokes, with an emphasis on stroke prevention.  Figure 1 demonstrates the lowered impacts of total serum and cholesterol level, lipids, overall fat percentage, and inflammatory responses, all of which contribute to issues like stroke.

### 1.1. Related Study

#### 1.1.1. Impact of Regular Walk and Physical Activity on Reducing the Chances of Stroke, CVDs, and Mental Health

According to the authors, the cumulative effect of the nutritional interventions investigated potentially lowered the risk of cardiovascular diseases by 12% and stroke by 11% [6]. This forecast is based on the assumption of nutritional improvements. It is estimated that one-third of all deaths because of strokes and heart attacks are caused by inadequate regular physical exercise [10]. Physical activity promotes endothelial function, which improves blood vessel vasodilation and vasomotor function [11]. Several studies have been conducted to explore the correlation between workouts and cardiovascular diseases in the ability to forecast stroke [12]. Exercise decreased the risk of overall heart diseases, sudden cardiac death, and stroke in a drug concentration pattern, according to a study of female invesigations [13]. There is a direct correlation between exercise programs and cardiovascular disease that is material up to a specific threshold of fitness, according to research. In the case of stroke, a similar relationship has been discovered. In [14], authors performed a study that included 15 peer groups and 5 case-control studies and found that people who are mildly active, highly active, and fit have a lower risk of stroke and mortality. It was observed that the people who are active, the significant decline in stroke occurrence was predicted to be around 20% to 27%. A concept of empirical evidence from the peer group and instance group studies that looked at the influence of workplace and relaxation workout on stroke risk found additional evidence in favor of exercise's preventive effect. The moderate levels of regular exercise at work were attributed to a 36% reduced risk of stroke when compared to being sedentary at the workplace [15].

#### 1.1.2. Impact of Alcohol on the Occurrences of Strokes

Various investigations have demonstrated a U- or J-shaped association between fatality and liquor use. The light or average drinkers die at a rate lower than those who do not drink, and those who excessively drink die at a greater rate [16]. Heavy drinkers had a greater risk of death from any cause and from pulmonary illness, particularly sudden cardiac arrest and blood clots. Excess liquor use can also contribute to mental, social, and physical problems [17].

#### 1.1.3. Psychosocial Factors That Can Reduce the Chances of Stroke and Mental Illness

Several social variables, including anxiety, stress, depression, social isolation, feelings of loneliness, and demanding work settings, have been demonstrated to be the major causes behind the development of stroke, cardiac diseases, and mental illnesses [18, 19]. If people can make their lives stress-free by adding a walking routine, then the chances of mental illnesses can be reduced remarkably.

#### 1.1.4. Blood Pressure Control Can Reduce the Chances of Stroke and CVDs

Hypertension is still the most significant contributing variable for both types of stroke attacks. High pressure of the blood is thought to be the cause of nearly 700,000 early deaths globally. It is a key risk factor for CVD and stroke. There is a strong and well-documented link between hypertension and stroke risk [20]. In healthy, normotensive persons, physical exercise is correlated with treating hypertension and a decreased likelihood of developing hypertension, thus changing a significant factor to stroke likelihood [21, 22].

#### 1.1.5. The Effect of Gender on the Chances of Occurrence of Strokes and Mental Illness

Physical activity lowered the likelihood of an acute stroke by 23 percent in women and 26 percent in men, according to a study of data from 35 prospective studies and 11 randomized controlled investigations on the impact of physical fitness on the stroke-related cause of death and disability. A potential peer group study of Women's Health Study participants [23] looked at the impact of different lifestyle elements on the risk of stroke in females and found a weak correlation between the risk of stroke and physical fitness alone. The literature reveals that combining routine exercise with smoking cessation, a low body mass index (BMI), a nutritious diet, and consuming alcohol in lower quantities was associated with a lower risk of stroke [8, 24, 25]. As many of the trials excluded females, there is less data on the function of exercise in improving the outcomes in females to make judgments and provide guidelines.

All these studies explore the impact of many factors on the occurrence of strokes, mental health, and CVDs. There is not a single piece of research work that can show the impact of walking on all these ailments. Hence, it has motivated us to conduct a study on the impact of walking on mental health and strokes. This paper explores the impact of walking on strokes, mental health, and CVDs using a research-based study. The research endeavors of the paper are mentioned below.

1. This paper attempts to highlight the impact of walking on human health, especially focusing on mental illness, CVDs, and strokes
2. To carry out this research, three groups of subjects are created, irrespective of gender. The subjects of the walking activity are divided into three groups, namely Group-1 walkers, Group-2 walkers, and Group-3 walkers
3. The activity of walking was derived based on the individual interests and ability to walk based on their physical fitness/health
4. All the participants were recommended to join Telegram and Kakao Talk Messenger to share their data routinely
5. The records are collected and analyzed based on the data collected from smart devices and mobile apps, along with the medical records shared by the participant subjects

The paper has four sections. The very next section provides highlights on the methodology used for this research study. The third section describes the results, and the final section summarizes the work.

## 2. Suggested Research Method

To meet the objectives of the proposed research study, we have designed an innovative method as described in this section. The study is supported by the physicians as the parameters considered for the study are suggested by physicians and health practitioners. The standardized parameters are considered for the proposed study based on the recommendations of physicians and healthcare practitioners. People remain active during their young age, which may be considered below 30, and as they get older, their physical activities start reducing, and health issues start emerging because of a sedentary lifestyle. In sports, military, and police department, people remain active for approximately 40 years, and in our study, we have taken the age group between 40 years and 55 years for measuring the impact of walking on human health and diseases, such as cardiovascular diseases and strokes. The research study is performed on 10,000 subjects between 40 years and 55 years of age. IoT (Internet of Things)- and AI-based smart devices are utilized to collect the data from the subjects. The data includes the medical problems of CVDs prior to the use of walking as daily exercise, and the data is collected after 90 days of walking routine.

It is important to motivate individuals who have earlier worked with the armed forces and individuals who were into sports to start with the regular walking routine along with the individuals who have worked in other sectors. The following steps have been carried out to inculcate the regular walking activity schedule of individuals for 90 days. The subjects have faced one or other cardiovascular diseases earlier and may likely have a stroke in the new future. The attempt was made to save them from strokes. A total of 4300 women and 5700 males have participated as subjects. For sampling, we have particularly focused on 40 plus people, whose participation in physical activities was almost zero because of their office and other engagements in life.

Below is the method devised to indoctrinate the habit of walking in the participants for 90 days.

1. To start with the activity, three groups of subjects are created, irrespective of gender. Telegram and another mobile app (KakaoTalk Messenger) are used to share the instructions for their participation.
2. The walking activity is divided into three groups, namely Group-1 walkers, Group-2 walkers, and Group-3 walkers.
3. Group-1 walkers have the plan for covering 6 miles in a week through a casual walk.
4. Group-2 walkers opt for the plan to cover 2 miles a day by opting for a casual walk but not a brisk walk.
5. Group-3 walkers opt for the plan to cover 3 miles in an hour or less than an hour in a day.
6. The liberty for walking was given based on individual interest and ability to walk based on their physical fitness/health.
7. All subjects were advised to join Telegram and Kakao Talk Messenger to share their data every day. The smartwatches used by people were GOQii Smart and Xiaomi. The data were also collected through mobile apps, such as YodoRun and Codoon.
8. The records are prepared based on the data collected from smart devices and mobile apps, along with the medical records shared by the participant subjects.
9. Other factors that are also studied along with the impact of walking on the participants are the hazardous impacts of smoking and alcohol consumption on cardiac and mental health.
10. The participants were segregated into three groups as per their choice of walking in kilometers.
11. The participating subjects are coached to be a part of the walking activity for 90 days. Walking was planned as per miles in a day or in a week.
12. All the participating subjects were allowed to share their data on Telegram and Kakao Talk Messenger.

The fields considered for research study are given below in Table 1.

By adopting the above method, an attempt is made to reduce the chances of cardiovascular diseases and strokes in the population aged between 40 years and 55 years. The next section elaborates the results and their respective interpretations.

## 3. Results and Interpretations

### 3.1. Impact of Walking on Alcohol Consumers with Respect to Strokes and CVDs

Patients of cardiovascular diseases who consume around 90 ml of alcohol every day or more than 90 ml on average are at a higher risk of having a stroke and other cardiovascular diseases. Alcohol consumption impacts liver function and raises blood pressure levels in the body, which indirectly induces the problems of cardiovascular diseases and increases the chances of stroke. In our sample population, there are 1800 alcoholic subjects who consume 90 ml or above alcohol on average every day. The reduction in the intake of alcohol to 60 ml from 90 ml and a regular walk of 30 minutes improved the health of subjects (sample population) remarkably and reduced the chances of having strokes by 20%. In this sample population, only males are considered who consume fixed amounts of alcohol every day. We have found it difficult to measure the changes. However, the impact of walking on health has been noticed well in the percentage scale for the occurrence of strokes in those who consume alcohol occasionally or in undetermined quantities. The facts are shown in Figure 2.

### 3.2. Impact of Walking on Improving Mental Health

In a sample population of 5000, the people are judged against the PSS and ESS scales. The values are obtained for 2000 participants who have opted for a casual walk for 2 miles a day, 1900 participants who have opted for 3 miles of brisk walk in an hour, and 1100 participants who have opted for a casual walk of 3 miles in a week. The PSS and ESS scores have improved remarkably for the participants who have taken an initiative to walk to improve their mental and physical health. Stress is also a major cause of mental illness and strokes. Improvements in the scorecards of PSS and ESS can certainly reduce the risk of CVDs and strokes. Group-1 represents casual walkers who walk 6 miles in a week, Group-2 shows casual walkers who walk 2 miles in a day, and Group-3 belongs to active participants who walk 3 miles every day in an hour or less. The scorecard is self-explanatory.  Figure 3 shows that Group-3 is the most beneficial group as its subjects are found to have improved PSS and ESS scores, while Group-2 is the next beneficiary. The third group (Group-1) also benefitted from the walk but not as much as Group-2 and Group-3, as shown in Figure 3. It depicts that walking not only reduces the chances of strokes but also improves mental health by reducing stress levels and by improving the sleeping score.

### 3.3. Improvement in Mood Swings after Regular Walk

In a population of 5000, 4100 people have been registered as unhappy with the problem of mood swings. A lack of confidence is also found to be a common problem among the participants. After participation in the regular and casual walk for 2 miles a day for 90 days, they found that their bad mood changed to a happy mood and the mood swings reduced remarkably. Besides, their confidence has increased as well The results are given in percentage, as shown in Figure 4. Based on the outcomes of the study, efforts are made to investigate the reasons behind mood swings and how walking has improved mood swings to alleviate the mental health of people aged between 45 years and 55 years. It was found that mood swings were common in women close to menopause, and walking helped them a lot in improving their mood and mental health. Even men get mood swings as they lose their confidence, as they are getting older.

The results presented in this section reveal that the 90-day walking program has created a good impact on the health of individuals by improving the physical and mental health.

### 3.4. Interpretations

The results presented in this section reveal that walking is certainly a solution for improving mental health as it minimizes mood swings, reduces stress levels, improves the sleeping index, and improves overall health. The PSS and ESS scores have improved significantly in the participants who have taken an initiative to walk for improving their mental and physical health. The results shown in Figure 4 depict that after participating in a regular and casual walk for 2 miles a day for 90 days, the participants have found their bad mood to have changed to a happy mood and their mood swings to have reduced significantly. In addition to it, the confidence is also alleviated of the participants. Group-1 comprises casual walkers who walk 6 miles in a week, Group-2 comprises casual walkers who walk 2 miles in a day, Group-3 comprises active participants who walk 3 miles every day in an hour or less. The scorecard is self-explanatory.  Figure 3 shows that Group-3 is the most benefited group as its participants have improved PSS and ESS scores. Group-2 is the next beneficiary. The third group (Group-1) is also benefitted from the walk but not as much as Group-2 and Group-3, as shown in Figure 3. It concludes that walking not only minimizes the chances of strokes but also improves mental health by reducing stress levels and by improving the sleeping score.

## 4. Conclusions

This paper presents a study on the impact of walking on strokes, mental health, and cardiovascular diseases. Mental health can certainly be improved by adding walking in the routine life, which eventually reduces stress, improves sleeping index, and improves the mental health of a person. The stress levels can be handled well by walking regularly, and a reduction in stress can lead to an improvement in mental health. It can be summarized that it is very important to be active after the age of 40 to get rid of physical and mental ailments. By changing their lifestyle and adding walking as a regular activity in life, individuals can control cardiovascular diseases and reduce their chances of having strokes. To conduct the research study, social media apps, such as Telegram and other fitness mobile apps, are used, as mentioned in the paper to record the data of the participants. The results show that individuals who even smoke and drink can improve their health by adding walking to their routine life. The scores of PSS and ESS are improved by 10% or more on average, which shows that people are able to reduce stress and improve their sleeping score by walking. Sound sleep is a must for avoiding strokes, improving mental health, and preventing cardiac diseases. The biomarker values are also recoded to prove the viability of the study, and the levels of CRP, P-selectin protein, and homocysteine are found to be improved, which shows that by adding walking exercise to one's routine, one can reduce the chances of having a stroke by 30% or more, depending on the routine followed by the individual. In the future, more parameters will be studied that can reduce the chances of having CVDs and strokes and improve the mental health of the individuals.

## Figures and Tables

**Figure 1:** Benefits of walking.

**Figure 2:** Walking impact on strokes as per the genders who smoke regularly.

**Figure 3:** Walking impact on stress levels to avoid strokes and improve mental health.

**Figure 4:** Walking impact on mood swings for better mental health.

**Table 1:** The parametric values taken for research study.

Attributes	Description
Subject_No	Each subject is given an ID
Group_id	Each subject is allocated a group ID
CVD_problem	This field mentions one CVD problem out of four types
History of strokes	This field contains bullion values in “yes” or “no”
Calorie chart	This field records calories burnt in a week after walking
C-reactive protein (CRP) initial	This field records CRP values before starting walking
Final_CRP	This field records CRP values after ending the walking routine after 90 days
PSS_initial	Perceived stress score is taken for study to check the stress levels of the participating subjects
PSS_final	The PSS of subjects was measured after 90 days of the walking routine
ESS_initial	Epworth sleepiness score is measured to check the stress levels before walking routine
ESS_final	ESS was measured again after the walking activity program of 90 days
Homocysteine_initial	Homocysteine levels depict the chances of having CVD or stroke, and this field records the initial levels of homocysteine before the participation of the subjects in the walking activity
Homocysteine_final	The final levels of homocysteine after the participation of subjects in the walking activity
P-selectin_initial	P-selectin protein measures are taken to see the chances of having strokes in the subjects
P-selectin_final	The levels of P-selectin are monitored to check the impact of walking activity
Walking_success	The field is used to record a bullion value in “Y” or “N,” where “Y” specifies that the program was successful and “N” specifies the inverse to it

## Data Availability

The data will be made available on request by the corresponding author.
